RETRACTED

# Energy Efficiency and Reliability Considerations in Wireless Body Area Networks: A Survey

**DOI:** 10.1155/2022/1090131

**Published:** 2022-01-17

**Authors:** Farman Ullah, M. Zahid Khan, Gulzar Mehmood, Muhammad Shuaib Qureshi, Muhammad Fayaz

**Affiliations:** ^1^Network Systems & Security Research Group (NSSRG), Department of Computer Science & Information Technology, University of Malakand, Chakdara, Dir (L), Khyber Pakhtunkhwa, Pakistan; ^2^Department of Computer Science, School of Arts & Sciences, University of Central Asia, Kyrgyzstan

## Abstract

In this paper, we have reviewed and presented a critical overview of “energy-efficient and reliable routing solutions” in the field of wireless body area networks (WBANs). In addition, we have theoretically analysed the importance of energy efficiency and reliability and how it affects the stability and lifetime of WBANs. WBAN is a type of wireless sensor network (WSN) that is unique, wherever energy-efficient operations are one of the prime challenges, because each sensor node operates on battery, and where an excessive amount of communication consumes more energy than perceiving. Moreover, timely and reliable data delivery is essential in all WBAN applications. Moreover, the most frequent types of energy-efficient routing protocols include crosslayer, thermal-aware, cluster-based, quality-of-service, and postural movement-based routing protocols. According to the literature review, clustering-based routing algorithms are the best choice for WBAhinwidth, and low memory WBAN, in terms of more computational overhead and complexity. Thus, the routing techniques used in WBAN should be capable of energy-efficient communication at desired reliability to ensure the improved stability period and network lifetime. Therefore, we have highlighted and critically analysed various performance issues of the existing “energy-efficient and reliable routing solutions” for WBANs. Furthermore, we identified and compiled a tabular representation of the reviewed solutions based on the most appropriate strategy and performance parameters for WBAN. Finally, concerning to reliability and energy efficiency in WBANs, we outlined a number of issues and challenges that needs further consideration while devising new solutions for clustered-based WBANs.

## 1. Introduction

In contemporary years, interest in uses of WBAN (wireless body area networks) and wearable technology has been remarkably boosted [1]. The number of patients, who need medical care by doctors/specialists are also increased as the increased of aging populations [2]. WBANs have been found to be the best and most cost-effective solutions for healthcare monitoring and related applications.

RETRACTED

WBAN is a network of low-power, nonhostile, smart, and compact sensor devices that can exchange their data over wireless media and operate in, on, or around a human's body [2]. It was once used to assess physical characteristics and maintain a record of any abnormal or critical circumstances in the entity body [3]. Among other characteristics electrocardiography (ECG) measures heart electrical activity, electroencephalography (EEG) measures brain electrical activity, and electromyography (EMG) is a type of sensor for determining the electrical activity of muscles. The data is subsequently transferred to a control device, such as a sink or gateway/PDA, where it is aggregated and nonaggregated (personal-digital assistant), and the acquired data can subsequently be communicated to remote monitoring destinations for diagnostic purposes [4, 5]. “WBAN is a subset of wireless sensor network (WSN)” [6]. In terms of employment, WBAN is divided into two types: *implanted WBAN* and *wearable WBAN* [7]. In “*implanted WBAN*,” the data from the implanted sensor nodes and the base station (BS) can be exchanged, while wearable devices and base stations (BS) can communicate their data with each other in “*wearable WBAN*” [8–10]. WBAN classifies each sensor into one of three categories: physiological, biokinetic, or environmental sensors [8]. Physiological sensors in WBANs, as depicted in Figure 1, are sensors that can assess corporeal phenomena/attributes such as temperature, blood pressure, and glucose monitoring. Biokinetic sensors are used to monitor and quantify human motion, such as calculating rotational angular rate and acceleration. Ambient sensors are any sensor that can measure environmental conditions, such as vibration, light, and pressure level. Environmental data is sometimes referred to as conservation data [11, 12].

Energy, processing, memory, and bandwidth are all limiting resources for WBAN. Instead of perceiving, sensor nodes waste a lot of energy while transferring data to each other. Furthermore, in most WBAN applications, changing or recharging batteries is not the best answer [13]. Because sensor nodes must be able to see and measure crucial active signs of human health, therefore, reliability is a critical concern. The key contribution of the proposed work is given as below:

- The proposed work effectively provides a critical analysis of energy efficiency and reliable solutions for WBANs
- This paper identifies various design and performance parameters that need careful consideration while devising any solution for WBAN applications
- Furthermore, research gaps are identified, and future directions are given to address these gaps in detail
- Finally, this research will help researchers to advance their understanding of the area of WBAN and the related challenges and current solutions of energy efficiency and reliability in WBANs

A set of most commonly used abbreviations and notations is given in Table 1.

RETRACTED

Section 2 explains the applications and architecture of WBAN.  Section 3 shows details about various unique characteristics and features of WBAN, while Section 4 shows the motivations towards the concepts of WBAN.  Section 5 explains the significance and importance of WBANs, while Section 6 explains the research issues and challenges in WBAN.  Section 7 describes the related work of the proposed solutions in the area of WBAN, and Section 8 discusses the limitations in the existing work.  Section 9 presents the conclusion.

## 2. Applications and Architecture of WBAN

WBANs have a wide range of uses, including medical and nonmedical applications. The basic purpose of all of these applications is to improve people's quality of life [14–16].

WBAN is a network that may be used to track personal health data such as heart rate and glucose levels, with the data being collected and stored on secure servers. Wearable and implantable medical applications are the two types of WBAN medical applications [2]. The following are some of the most well-known wearable medical applications of WBANs:

- Sleep staging: sleep is a regular physiological function and behaviour in our daily lives [17]. WBAN was used to track sleep disorders. Sleep deprivation has been linked to an increased risk of heart disease. Drowsiness at work and drowsy driving are also monitored because a big percentage of the population suffers from sleep disorders
- Asthma: WBANs are utilised to monitor asthmatic patients since they can provide a real-time reaction to a surgeon by screening for sensitising substances in the air
- In sports: WBAN analyses player's performance by measuring fatigue levels using glucose, temperature, and heart rate sensors. In fact, WBAN is utilised to scrutinise a player's training regimen, including motion capture and rehabilitation [18]
- In a battlefield: soldiers are equipped with WBAN-based sensors that alert commanders to their motions, such as running, digging, and shooting

The phrase “implanted WBAN” refers to nodes that have been implanted into the human body and are most typically used in diabetes and cardiovascular monitoring. Similarly, WBAN sensors can sense cancer cells throughout the body and send a real-time reaction to healthcare user for diagnostic purposes [2].

WBAN is utilized in the following industries for nonmedical purposes.

- In the entertainment sector: in computer games and gesture detection, body sensors are used. These networks are used for real-time streaming, such as audio and video [2]. WBAN is used for amusement and social networking, as it includes an MP3 player, camera, and microphone
- In a consumer electronics sector: body sensors are sensors that are affixed to a person's body and are used to send and communicate information to devices, i.e., a music player, headphones, a cell phone, and hearing aids [2]
- Off-body: sensors are used to monitor and identify nonmedical situations in the home, such as fire and toxic gas, and then transfer this information to sensors linked to the body [2]
- “In lifestyle sector”: WBAN is a technology that can be used to recognise a person, recognise their individual data, and pinpoint their particular position [2]. It has been used to detect emotions such as fright, respiration rate, and pulse rate. It aids in the detection of posture and ambient intelligence
- In aerospace: WBAN used to employ a flying system to warn the pilot in the event of an emergency or other urgent circumstance by gathering data from many sensors [2]

The data requirements vary according to the different sorts of applications. When it comes to bit error rate (BER), the reliability of the conveyed data is based on the corrected data to be given to healthcare experts (BER). Applications with a low data rate have a high BER, while those with a high data rate have a lower BER [13]. The most important design concern, as discussed in the following sections, is reducing energy use. During sensing, processing, and communication, energy is consumed. Depending on utility, shape, and location, different applications and their basic requirements require different amounts of energy. Furthermore, providing QoS needs in medical healthcare apps is critical [19]. All these requirements associated with different categories of applications are tabulated in Table 2.

RETRACTED

Architecture of WBAN: WBAN, from an architectural aspect, comprises of low-power sensing devices that are positioned inside or externally but are not confined to the body; in fact, WBAN has been employed in a wide range of applications, including entertainment, consumer electronics, and lifestyle. Almost every WBAN application has a three-tier architecture system as shown in Figure 2 [20].

Different sensors are utilised to analyse physiological parameters and their activities in, on, or around the human body. The data then communicated to the personal server (PS) in tier 1—also branded as intra-WBAN communication (PDA). Tier 2 communication is also recognized as inter-WBAN communication and occurs between a PS and access points. The goal of tier 2 communication is to join WBAN to a variety of systems that may be accessed easily in our daily lives, such as the Internet and cellphone networks. PDA or gateway was used as a link between layer 2 and this tier; i.e., in some applications from the Internet to the medical server in tier 3, known as beyond-WBAN communication (MS). One of the most important components is a database in tier 3 communication that stores user's profile and medical history. As a result, the emergency can be communicated to the patient or physicians via SMS (short message service) or the Internet. In WBAN communication, there are several different operational scenarios:

- Implant to implant
- Implant to body surface
- Body surface to body surface
- Body surface to external

Requirements of WBANs: WBAN creation, however, is a difficult process due to the wide range of needs. The most essential IEEE TG6 requirements are discussed in this part, and some are discussed in the following sections [21]. We will go through some of the general criteria for various types of WBAN applications in this section. As indicated in Table 2, we examine bit rate, BER, and latency requirements in particular. Depending on the application and the type of data, different bit rates are necessary. BER is also discussed for a variety of applications in Table 3. Another crucial component is the end-to-end delay. Varied types of traffic have different priority levels, for example, emergency traffic requires a minimum wait.

## 3. Unique Characteristics of WBAN

WBANs, unlike WSNs and ad hoc networks, are a specific breed of WSN with their own set of characteristics. WBAN is typically placed in or on a human body and is utilised for healthcare purposes. As a result, design issues such as compactness, compatibility, and inconspicuous deployment are critical. The following are some of the distinctive qualities that present WBAN researchers with new technical challenges:

- Architecture of node: based on its functionality, implementation, and role, each device/node in the WBAN can be classified into three groups [8]. Nodes are classified as personal devices (PDs), sensors, or actuators based on their functionality [2]. Nodes can be categorised as implant devices, body surface devices, or external devices depending on how they are implemented. Each node in the WBAN is classified as a coordinator/controller, end node, or relay node, depending on their function. Maintaining battery power at the sensor node is crucial since each sensor device used in WBAN must be noninvasive, compact, and pleasant, as well as invisible [22]
- Node temperature increase: because of communication radiations and circuitry power loss, the temperature of sensor nodes in WBAN may rise [23]. As a result, SAR (specific absorption ratio) must be considered when developing any WBAN application [24]
- Node density: the total number of devices in WBAN might range from a few sensors or actuators to tens of thousands of sensors or actuators. Unlike WSN, WBAN has a low density, sparsely placed nodes, and decreased node redundancy [25]
- Reliability and security: in WBAN, each sensor-device may sense and monitor a patient's personal and important data [10]. As a result, it is necessary for monitoring data to be provided in a fast, accurate, and secure manner
- Mobility: the same pattern of mobility will be share by WBAN nodes as the user may move around [25]. Design consideration contains the packaging and placement of sensor nodes
- Cost-efficient: sensors and equipment utilised in WBAN are inexpensive and readily available in consumer electronics applications [26]
- Topology of the network: there are two types of network topologies utilised in resource-constrained WBAN: star and hybrid mesh topology [27]. However, it is extremely desirable to create or build a reduced topology in all WBAN applications in order to save energy while maintaining crucial network characteristics such as connection and coverage

RETRACTED

## 4. Motivations towards the Concepts of WBAN

In the medical area, WBAN is a critical tool for patients who do not have access to doctors or who are experiencing difficulties owing to age, time, distance, hospitalisation costs, injuries, or disability. The majority of hospitals are also experiencing difficulties due to a lack of doctors. The following are some of them:

- For distance doctors who are unable to keep track of their patients
- Physical visits to the doctor for patient monitoring take time
- Elders are unable to make timely visits to doctor's clinic
- It is tough for doctors to keep track of patients during casualties (e.g., wars, Earth Quick)
- Disabled persons have a difficult time going to the doctor

Other issues include a lack of doctors and suitable equipment due to limited or nonexistent funding, as well as a scarcity of educated professionals to diagnose patients' illnesses in hospitals.

## 5. Significance and Importance of WBAN

The concept of WBAN is one of the solutions to all of these issues. The WBAN is beneficial since patients may require assistance at times.

- Continuous patient monitoring
- Lowering hospitalisation costs
- Lowering the rate of untimely deaths
- Improving health-care efficiency through communication technology
- Emerging medical care
- Addressing transportation issues
- Patient mobility issues
- Emergency care for injuries sustained in traffic accidents

In hospitals, patient monitoring is the most important responsibility for doctors to conduct. The WBAN is a new technology that is being utilised to monitor patients. Doctors are sometimes unable to supervise patients because to a variety of factors, including casualties (wars, earth rapid assaults), patient's age, disability, and hospitalisation costs. The WBAN has been shown to be a good substitute for or precursor to patient monitoring at home. It has significant advantages, particularly for the disabled and elderly patients who can be monitored remotely from anywhere at any time. The WBAN provides assistance to patients at no cost and without causing any mishaps. As a result, the usage of WBAN in the medical area for patient facilitation and monitoring has become popular.

RETRACTED

## 6. Research Issues and Challenges in WBAN

WBAN's rapid growth has posed considerable hurdles for the research community despite the fact that it has a wide range of applications and benefits. Some of the most important WBAN research issues and difficulties are listed below.

### 6.1. Network Topology and Energy Holes

WBANs' overall performance and energy consumption are influenced by their network topology [6]. A good network architecture is critical in WBAN due to body postural movements, poor transmission range, energy restrictions, and the different type of sensor nodes. The majority of research placed important data monitoring sensor nodes near the BS (base station), which employs single-hop communication, whereas normal data monitoring nodes further away used multiple hop communication [28]. When the demand on a sensor node is spread unevenly, node's energy is quickly depleted, resulting in an energy hole [29]. In order to prevent energy and coverage gaps, the deployment of nodes is a vital step in the WBAN process. When there is a coverage hole, the area under that node's observations is unsensed. The problem of energy holes can be addressed by establishing efficient criteria for selecting forwarder/leader nodes and communication protocols.

### 6.2. Energy Efficiency and Network Lifetime

Each sensor in the WBAN system has its own energy, memory, computation, and bandwidth constraints [30]. When sensor nodes exchange their data with each other rather than sensing, a large amount of energy is consumed, and due to the nature and operational limits of the application, recharging or replacing batteries is neither practicable nor desirable [31, 32]. A forwarder (FWD) node's transmission energy can be computed as:

(1) ETxFWD= N´.£.ETxP‵,đ+ N´.P‵.£.ETx‐proc,

where “£” is the data aggregation factor, “$\overset{`}{N}$” denotes the total number of nodes,“*Ῥ*” indicates the size of the packet, and “*đ*” is the distance between forwarder nodes, and sink is denoted by this value. ETx and ERx indicate the transmitter and receiver's per-packet energy consumption expenses. ETx-proc and ERx-proc are the energy necessary to run the electrical circuits of the transmitter and receiver, respectively. So, in terms of total network lifespan, a forwarder node's total transmit energy may simply be calculated as:

(2) $$\begin{array}{c} {E_{\text{Tx}}}^{\text{NLT}}=\int^{t.}{E_{\text{Tx}}}^{\text{FWD}}dt. \end{array}$$

As a result, in WBAN, energy-efficient solutions are required to increase network's stability period, and, as a result, its enhance network lifetime [33].

RETRACTED

The total duration of network activities until an end node is depleted is referred to as the network lifetime [1, 28, 29]. The network lifetime is an essential feature that directly affects network's throughput. The total number of successfully received packets is referred to as network throughput. With a longer network lifetime, throughput is maximised [1, 28, 29].

### 6.3. Stability Period and Reliability of Network

The time between the start of operations and the expiry of the first sensor node is known as network's stability period [1, 29]. Network's stability period is critical since we require uninterrupted functioning for days, if not weeks, without operator intervention; thus, we must reduce communication. As a result, a load balancing strategy must be proposed in which the load is spread uniformly or evenly among sensor nodes.

The term “reliability” refers to the fact that health-care practitioners receive monitoring data in a timely and accurate manner [28, 34]. WBAN sensors must be capable of viewing and detecting essential active signs of human health; therefore, reliability is critical [35]. WBAN sensors must be capable of viewing and detecting essential active signs of human health; therefore, reliability is critical [2, 36].

### 6.4. Fault Tolerance

In WBAN, fault tolerance is also an important issue, which means that how to maintain network operations without faults and failures, and recover failed nodes. In a resource constrained WBANs, fault-tolerance is highly important because the deployed sensors are battery operated and have a limited battery lifetime [37]. Faults can be divided into three categories: i.e., faults were caused by nodes, sinks, or network issues [38]. The main causes of node failure are hardware (sensing, processing, memory, transceiver, and battery) and software (MAC, application, and routing) [39]. Network faults can arise because WBAN applications are responsible for the delivery of collecting information from sensor nodes towards the sink. Routes or link failures can occur due to the interference in the link or collision of packets. Fault tolerance in WBAN can be performed in a variety of ways; cooperative communication and network coding, on the other hand, are two effective strategies for improving network fault tolerance and reliability [40]. Similarly, fault tolerance techniques are necessary to overcome sink failure, because the sink is a critical component of WBAN, and its failure will result in the entire network failing.

RETRACTED

### 6.5. Compatibility Issue and Unobtrusive Deployment

To provide plug and play collaboration among sensors and to promote a reliable exchange of information, WBAN system ensures tights or smooth data transmission across different standards [2] such as Bluetooth and ZigBee. Therefore, the challenge is to design a WBAN that requires an unassuming placement of sensors. Such solutions must be lightweight and nondisturbing, which would not change or disturb daily routine of the user [41].

### 6.6. Usability and Interoperability

WBANs must have the capability of self-configuration and self-maintenance because medical staff will set up WBAN instead of ICT (Information and Communication Technology) engineer. When a sensor is placed on the body and turned on, it must be able to connect a network and determine the structure of routes without interference from the outside world [36]. When new services are added to a network, it should be capable of reconfiguring itself [6]. Moreover, an alternate path should be set up, when one path fails.

Relying on the kinds of application, WBAN applications can be wearable on the surface of the body and also can be implanted inside the body [8]. These devices, hence, can operate in dissimilar frequency bands and PHYSICAL layers (PHYs). Thus, the WBAN applications must be interoperable at multiple frequency bands and support multiple PHYs.

### 6.7. Security

WBAN sensor nodes collect sensitive personal information, making it subject to active and passive attacks including eavesdropping, spoofing, and snooping. Because the WBAN network allows several users to transmit and receive data, it is vital that the data be allowed to be exchanged. Information/messages must also be nonrepudiated, as repudiation happens when the sender and receiver deny that messages were transmitted and received. As a result, multiple sorts of security criteria are required to tackle security concerns, authentication, privacy, data consistency, data freshness, availability, and secure localization are just a few examples [2]. Moreover, established cryptography security techniques are employed to satisfy WBAN's basic security needs. However, due to the resource limits imposed by WBANs, such solutions should be computationally processing light [42–44].

RETRACTED

### 6.8. Scalability

In the design of routing protocols for WBAN, scalability is also an important element to be considered in the application development. Scalability refers to a network's ability to add or remove devices without causing significant changes to network's structure or operations [31]. To put it another way, the protocol should be scalable and flexible to numerous alterations that may occur in WBAN owing to the addition of additional sensor devices from time to time [45].

## 7. Literature Review

We have covered several research issues and challenges related to the field of WBAN in the previous section, which shows that energy efficiency, reliability, and network stability period are the most vital issues in WBAN. Although much study has been done on these topics, it is still required to propose more stringent energy-efficient and reliable approaches to extend the lifetime of WBANs while keeping in mind their resource constraints. In this section, we review the most notable WBAN activities in the domain of energy efficiency and reliability, as well as the most relevant-related work.

We analysed the existing procedures and schemes critically and summarised their strengths and weaknesses. Because each sensor is battery powered, and a lot of energy is spent on communication rather than sensing, recharging or replacing batteries is a major difficulty in WBAN [41, 46, 47]. To reduce energy, WBAN routing algorithms include single-hop and multihop strategies. In a single-hop approach, a sensor node transfers sensitive data directly to the PS. Single-hop communication is ideal for sensors situated close to the sink; however, because nodes located further away from the sink use more energy while transmitting packets to the sink, this method is ineffective. A forwarder node in multihop communication transfers data from other nodes while saving energy consumption of the network [48]. In a multihop strategy, however, nodes closer to a sink become a hotspot as a result of relaying data from other nodes [41, 49].

Furthermore, the most common types of routing protocols comprise cluster-based, crosslayer, thermal-aware, quality-of-service, and postural movement-based routing protocols [16, 50]. In this study, we have focused on the first three techniques, which serve as a foundation for the other two approaches as depicted in Figure 3. These are main category of routing protocols in WBANs.

### 7.1. Crosslayer Routing

The crosslayer routing is a protocol stack used in WBANs that incorporates two or more levels to improve efficiency and interoperability between techniques/protocols. This category includes Braem et al. [51] proposed a Wireless Autonomous Spanning Tree Protocol (WASP) which is built on a spanning tree structure in which a time axis is separated into slots. Sensor nodes establish a link by telling their offspring nodes, and each node is assigned an isolated WASP-scheme message. However, poor link quality and routing overhead are protocol's principal drawbacks, as WASP lacks a data concatenation method for reducing the amount of transfers. To improve the WASP, Braem et al. [52] suggested a Cascading Information of Controlling Access and Distributed Slot Assignment (CICADA) protocol for WBAN that uses Time Division Multiple Access (TDMA) with two-way communication capability. It uses a data-gathering tree to manage data transfer. For data transfer to its parent node, each CICADA node calculates two parameters. To begin, figure out how many slots the parent node needs to receive all data from its child node. Second, before delivering data to the parent node, the child node determines how many slots are available. Unlike WASP, CICADA is a low-energy, high-reliability protocol that maximises throughput while reducing data loss. The authors, on the other hand, do not address the issues of poor link quality, mobility, load balancing, and routing overhead. Furthermore, the performance of the CICADA protocol declines dramatically throughout the sink to sensor-node transmission. In [53], it is intended to use the Time-Zone Coordinated Sleeping Scheme (TICOSS). By defining the shortest travel route to the WBAN coordinator, TICOSS improves the IEEE 802.15.4 standard by controlling all sensor nodes as Full Functional Devices (FDD). As a result of the V-scheduling, the sensor node's energy is preserved while concealed terminal collisions are minimised. Moreover, this method allows IEEE 802.15.4 to support mobility while also doubling its operational lifetime in high-traffic environments. BIOCOMM [54] is a crosslayer routing protocol for WBANs that combines the network and MAC layers to improve overall network performance. In [55], Adaptive Multihop Tree-Based Routing (AMR) is a distributed spanning-tree system that considers battery level, Received Signal Strength Indicator (RSSI), and hop count. AMR distributes energy consumption evenly among sensor nodes, resulting in a longer network lifetime and more transmissions per packet delivered. However, extrapacket switching between sensor nodes is necessary.

RETRACTED

### 7.2. Thermal-Aware Routing

In vivo sensors can be implanted inside the body, and WBANs with hot-spot monitoring are a major feature. The temperature of sensor nodes rises and thus heats up in multihop methods due to processing, communication radiation, and circuitry power consumptions, which might damage human tissues and compress blood flow. As a result, a thermally aware procedure is required, which can reduce energy usage while extending the stability period.

Tang et al. [56] TARA is a thermally aware method that was proposed (Thermal-Aware Routing Algorithm). When all which surrounds adjacent nodes are hot spot excluding the sender node, the sender node will select other paths in TARA. TARA receives these hotspot nodes as a fresh candidate for later routing after their temperatures drop below a certain threshold. However, greater packet transmission latency (latency), bandwidth waste, and energy consumption are all disadvantages of this method, making it unsuitable for WBANs. Bag et al. [57] introduced LTR (less-temperature rise), a thermally aware routing protocol based entirely on a greedy approach. It delivers data to nearby sensors with the lowest temperature for its rating, unlike TARA. Although because packets are travelling via paths that may or may not lead to the destination, this approach has disadvantages such as greater packet transmission delay (latency), bandwidth waste, and energy usage. However, to enhance LTR, Bag et al. [57] developed ALTR (adaptive less-temperature rise), a thermally aware routing protocol analogous to LTR. Disparate of LTR, when the number of hops surpasses a base threshold, Max Hop Adaptive can employ shortest hop routing (SHR) as a backup means of sending data as quickly as possible. The disadvantages of this method, like LTR, are increased energy consumption and a higher rate of packet loss.

Takahashi et al. [58] introduced the LTRT (least total route temperature) thermal conscious routing approach, which addresses the shortcomings of TARA, LTR, and ALTR. LTRT is a hybrid protocol that combines the LTR and SHR protocols (shortest hop routing). Among all possible packet delivery routes, it chooses a lower-temperature path from the source to the destination. By lowering the amount of hop counts, LTRT prevents wasting network capacity. The main disadvantage of this strategy is operational overhead, since it requires relaying a sensor's temperature state across sensor-nodes, which raises temperature and hence increases battery consumption. Javaid et al. [23] suggested M-ATTEMPT (Mobility Supporting Adaptive Threshold-Based Thermal-Aware Energy-Efficient Multihop Protocol), a well-known thermally aware routing protocol. Data must be directed away from sensor nodes capable of tracing/sensing connection hotspots in this fashion. Among the numerous accessible options, the shortest path is chosen. When there are multiple routes with the same number of hops, the one with the least amount of energy depletion is chosen. A joint-invitation request is sent if a sensor node moves during a data collection cycle, and a joint-request is allowed if the number of subnodes is less than three when checking the child nodes list of a parent. When sensor nodes detect a connection hotspot, packets are forwarded via a long alternate path, resulting in higher energy usage. Despite its benefits, when a sensor fails in M-ATTEMPT, there is no other option. Furthermore, instead of being situated based on their energy level, the location of these sensor nodes is determined by their data rate. To handle the drawbacks of “M-ATTEMPT”, Ahmad et al. [59] developed the notion of “RE-ATTEMPT,” a thermally unaware routing strategy “Reliability-Enhanced Adaptive Threshold-Based Thermal Unaware Energy-Efficient Multihop Protocol (RE-ATTEMPT).” RE-ATTEMPT employs a multihop communication paradigm in which the shortest route between sensors and sink nodes is selected. In this approach, sensor nodes exchange HELLO messages to discover all accessible routes. When a current path is unavailable, it chooses a less-than-ideal alternative to ensure reliable transmission. Because of limited number of forwarder nodes, this strategy can avoid relaying of unnecessary traffic. On the other hand, direct communication with the sink is not the best solution for attaining low latency at the expense of energy and reliability since it increases the risk of packet loss due to long-distance communication [60].

RETRACTED

Multimode Energy-Efficient Multihop Protocol was proposed (M^2^E^2^) by Rafatkhah and Lighvan [61]. For WBANs, M^2^E^2^ is a high-throughput, energy-efficient, and reliable routing system. It solves flaws in the M-ATTEMPT protocol, such as when the parent node refuses to accept a request from a moving node that is also a parent node. However, no effective method for mobility support has been provided, and there is still no alternate mechanism for sending packets to destinations after a node dies.

### 7.3. Cluster-Based Routing

These solutions are the best way for WBANs to address the issues in the above-mentioned schemes. In a cluster-based routing system, data is transferred to the base station through cluster heads in their respective time slots, which decreases energy drinking and hence enhances stability period. In addition, cluster-based strategies are used to extend the life of the network by decreasing energy consumption. So, Braem et al. [62] presented “relaying and cooperation techniques,” a dedicated relay sensor nodes collaborate in the network. This technique extends the life of the network by balancing energy usage across sensor nodes to maximise throughput. However, on the other hand, this paper did not go into great depth regarding where to put the relay node or how to choose it. In addition, the delay and packet loss ratio must be considered.

RETRACTED

In WBANs, Ehyaie et al. [63] suggested a relay network concept, which is a set of multiple relay nodes scattered throughout the human body that works as a WBAN transport network. With the use of a dynamic routing algorithm, the suggested approach increases reliability by providing many paths for communication from each sensor to the sink. When the sensor node and sink are not in range of one other, a relay network is the ideal option for NLOS (“Non-Line of Sight) communication”). In terms of mobility assistance, this system is effective. However, employing a relay network to analyse latency and packet loss ratio is critical.

“SIMPLE (Stable Increased Throughput Multihop Protocol for Link Efficiency)” is an energy-efficient routing protocol suggested by Nadeem et al. [28]. In SIMPLE, the minimum function is utilised to select a forwarder node. In each round, the forwarder nodes with the highest residual energy and the shortest distance to the sink node are selected. In SIMPLE, the energy depletion across sensor nodes is balanced by residual energy parameter while the distance value provides maximum throughput. This technique has a longer network lifetime, a longer stability period, and a higher throughput than the M-ATTEMPT protocol. The criterion for selecting a forwarder node, however, is unsuccessful since traffic load is not properly spread among sensor nodes. Furthermore, due to frequent data transfer, the SIMPLE protocol's performance worsens in crucial data reporting-based applications because it does not compare current sensed value to previously detected value. To address the shortcomings in the SIMPLE protocol, Javaid et al. [1] suggested the “IM-SIMPLE (Improved Stable Increased Throughput Multihop Protocol for Link Efficiency)” for WBAN. The IM-SIMPLE scheme major purpose was to handle mobility. In addition, to maximise throughput, a linear programming approach is implemented. For standard sensor nodes, IM-SIMPLE employs a multihop communication mechanism to save energy. A sink node can also choose a forwarder node with the lowest cost function using the TDMA scheduling technique, and all other nodes can send data to the forwarder node in their allowed time slot. One of scheme's significant drawbacks is the forwarder node's poor selection criterion. Because, a forwarder node closer to the sink is frequently picked, therefore, the energy of such nodes reduces quickly, and they expire quickly. In addition, given that the link quality and the path loss are not much considered in IM-SIMPLE protocol, therefore, the number or percentage of dropped packets in a given period is greater than that for SIMPLE [64]. To increase energy efficiency and reliability in WBANs, Sandhu et al. [65] have designed the “FEEL (Forwarding Energy-Efficient Data with Load Balancing) protocol” to improve energy efficiency and reliability in WBANs. FEEL is an energy-efficient protocol because it efficiently uses the battery power to provide network stability for a longer period of time, because effective criteria for the forwarder node selection is determined as compared with protocols such as SIMPLE and IM-SIMPLE. Throughput and network longevity are increased as a result of this excellent forwarder node selection. However, in the event of a path failure, the retransmission of data packets receives less attention [66]. Ullah et al. [67] present a novel “Energy-Efficient and Reliable Routing Scheme (ERRS)” to improve WBAN resource-controlled network stability and reliability. Selection of forwarder node and rotation of forwarder node are two unique ERRS solutions. The suggested ERRS uses adaptive static clustering technology to improve network life and stability, leading to greater reliability. The proposed ERRS proved to be a WBAN routing solution that is effective and reliable. But the basic problem of scalability and mobility will also be tackled in our future research work in order to deal with the wide range of prospective WBAN applications. For instance, it is fascinating to examine the impact of different human body components, on the overall stability and the network lifetime of WBANs.

RETRACTED

### 7.4. QoS-Aware Routing

Quality of service (QoS) is the essential factor of all applications within WBAN. QoS provisioning for WBAN is a key issue due to considerable challenges and the critical nature of data in many applications. Various types of traffic in WBANs have different QoS needs [68–71]. The following paragraph discusses some of the most important approaches for QoS-aware routing.

The “Data-Centric Multiobjective QoS-based Routing protocol” is introduced by Razzaque et al. [72] which is known as (DMQoS). The proposed protocol's goal is to use a modular architecture to enable different channels for packet delivery based on data priority. It is made up of five modules, one of which is dynamic packet classifier dividing data into four categories (ordinary, delay sensitive, critical, and reliability sensitive packets). In terms of energy economy, average latency, and reliability, the proposed approach improves performance. However, the suggested protocol increases traffic load, causing network congestion and compromising end-to-end latency and reliability.

RETRACTED

Khan et al. [73, 74] suggested a delay-sensitive data QoS-aware routing technique termed as (QPRD). This protocol is an evolution of the energy-aware peering routing (EPR) protocol, which divides receiving packets into two groups: conventional packets and delay-sensitive packets. The proposed protocol devises a technique for determining the optimum route for both types of packets while taking into account QoS requirements. This protocol is made up of seven modules: the QoS-aware queuing module receives and sends incoming packets into two queues based on their kinds, which operate on a first-in-first-out basis. QPRD performs admirably with regard to the packet delivery and network load.

Monowar et al. [75] presented a WBAN-specific “thermal-aware multiconstrained intrabody QoS routing protocol” called “TMQoS.” The main aim of the suggested approach is for the QoS requirements of various applications to be fulfilled while the sensor node temperature is taken into account. For routing table building, the proposed protocol makes use of the crosslayer routing architecture. There are ten modules in this technique. The arriving packets are divided into four types by a QoS-aware packet classifier. TMQoS meets the QoS standards with lower latency and improved reliability. On the other hand, the TMQoS strategy fails to balance energy utilisation between sensor nodes. In addition, the single-hop approach cannot always ensure the necessary delay and reliability in such a setting. Bangash et al. [76] proposed a “Critical Data Routing (CDR)” for WBAN in a similar way. The suggested protocol's goal is to discover the optimum path for essential data. To improve reliability, essential data must be transmitted in a short amount of time. The paper addresses difficulties caused by postural movement within the human body and by path loss and an increase in the temperature. The proposed CDR protocol met its goal of reliably delivering essential packets within a specified time limit. The recommended strategy, on the other hand, performs poorly in terms of average temperature rise.

In Tauqir et al. [14], “Distance-Aware Relaying Energy-Efficient System (DARE) was presented as an energy-efficient and high-throughput clustered-based routing protocol for WBANs.” Eight patients in a medical unit were observed using DARE by evaluating several sink placement scenarios. Seven sensor nodes with infinite energy resources, including one relay node on the chest and one main sensor on the bed, were deployed/attached to every patient. The propagation latency in DARE is found to be comparatively high. Furthermore, the link quality, path loss, and cost of the network were not adequately addressed [77].

RETRACTED

“Linked-Aware Energy-Efficient Routing Protocol (LAEEBA)” is an “energy-efficient link aware routing system for WBAN” presented in [78]. LAEEBA has proven to be a reliable scheme with low path loss and a high total network performance. Furthermore, employing both single-hop and multihop communications, the network lifetime is increased, reducing the consequences of path-loss. Furthermore, LAEEBA uses the same forwarder node selection criteria as the SIMPLE protocol, which has been shown to be effective in terms of energy efficiency and network stability. However, the fundamental disadvantage of this protocol is that data packets have a higher overhead during data exchange [64].

To address the shortcomings of LAEEBA, Ahmed et al. [79] suggested “CO-LAEEBA (Cooperative Linked-Aware Energy-Efficient Routing Protocol for WBAN),” based on a cooperative multicasting technique. Two or more pathways exist in CO-LAEEBA, and critical data is transmitted through single-hop communication while normal data is transmitted through relay nodes (a node which acted as a cooperative node). When a sensor node's remaining energy exceeds that of a relay node, packets are routed directly to the sink. When a sensor node's remaining energy is less than that of a relay node, it uses multihop communication. The CO-LAEEBA simulation results show that it enhance the existing protocols in terms of maximum throughput and network lifetime. However, as the CO-LAEEBA protocol uses only a small number of forwarder nodes, too many links for data packet transmission from source to destination are also required [64].

### 7.5. Postural Movement-Based Routing

The topology of the network is affected by body movements, link failure, and environmental impediments, causing linkages to disconnect. Many researchers have addressed this issue, and a cost function has been created to identify the best method to forward packets to the sink on a periodic basis. A few of the protocols that fall within this category are listed below.

In Quwaider and Biswas [80], on-body store and flood routing (OBSFR) is proposed on-body packet routing technique for wireless body area networks (WBANs) that provides improved routing time and hop count. The proposed protocol employs an opportunistic forwarding strategy depending on node distance from the on-body sink node. Furthermore, the end-to-end packet delay, number of packets per transmission, and packet delivery ratio are checked and compared to existing routing protocols. Quwaider and Biswas [81] proposed DTN routing in a wireless body area network (WBAN), taking into account a dynamic postural splitting technique called as distance vector with postural link cost (DVRPLC). A prototype WBAN has been built in the proposed work to test body topology disconnections in the presence of short-range radio links and human postural mobility. This protocol's major purpose is to reduce end-to-end delay. The average latency, packet delivery ratio, and packet hop count are all measured. In comparison to existing probabilistic, opportunistic, and utility-based DTN routing protocols, the output results suggest that the proposed approach can deliver better outcomes. Maskooki et al. [82] In WBAN, an opportunistic routing scheme was developed to improve the network lifetime by using the movement of body components. The proposed approach's major goal is to reduce end-to-end delay. The proposed strategy outperforms the other single-hop and multihop strategies in terms of performance. The average energy usage per bit is kept as low as possible. While in Movassaghi et al. [83], ETPA (energy-efficient, thermal, and power-aware routing) protocol was designed to lower node temperature and prevent hotspot development. For the cost function calculation, ETPA took into account the node temperature, energy level, and power gain. The proposed protocol effectively exploited the available resources in WBAN routing protocols, according to the performance study. Many energy-efficient and reliable routing algorithms advise boosting network stability and reducing delay; however, during the network implementation, network organisation, and internode communication stages, less attention has been paid to energy saving and higher reliability. The load is not spread evenly among sensor nodes because the forwarder node selection criteria and the appropriate number of relay nodes are inefficient [84]. As a result, in order to improve WBAN's stability period, an energy-efficient and reliable routing approach is necessary.

RETRACTED

## 8. Discussion

The previous section described and critically analysed existing energy-efficient and reliable routing protocols, such as crosslayer, temperature-aware, and clustered-based techniques. Crosslayer routing approaches are inadequate for WBAN because loads are not equally distributed among sensor nodes. This increases the odds of an energy hole. Because of the high computational cost and complexity, it is not suited for energy-constrained, low-processing, low-bandwidth, and low-memory sensor-nodes. For implanted WBAN, thermal-based techniques are required. However, in wearable WBAN, detecting hotspot nodes has a higher overhead and consumes a lot of energy. We have identified and stated the following most relevant design and performance parameters for WBANs, keeping in mind the resource-constrained nature of WBANs and based on a rigorous examination of state-of-the-art systems. When creating and testing new energy-efficient and reliable WBAN systems, these crucial parameters should be taken into account.

### 8.1. No. of Dead Nodes

This metric shows the total number of nodes whose remaining energy has been completely exhausted. The number of dead nodes is reduced when load is distributed consistently or evenly among sensor nodes, and vice versa, resulting in increased network lifetime.

### 8.2. Packets Sent to Sink

The total number of packets sent to the base station or sink is indicated by this parameter. The number of packets sent to the sink is proportional to the total number of nodes that are alive. The total number of packets transferred also depends on whether the WBAN application is time-driven or event-driven.

### 8.3. Packet Dropped Ratio

This indicator represents the total number of dropped packets as a proportion of the total number of sent packets. The number of transmissions is proportional to the number of packets discarded. The random uniform model is used to calculate packet dropped ratio. A communication link's status can be excellent or bad depending on the likelihood, with 0.7 being a favourable link status probability.

### 8.4. Packets Received at Sink

This metric represents the total number of packets successfully received at the sink. WBANs are designed to receive as much data as feasible while discarding as few packets as possible at the sink. As a result, because WBANs can monitor any type of abnormal state in the patient, the sensing data must be collected precisely at the sink.

### 8.5. Stability Period

Stability Period refers to the period of network activities from the start of the established network until the expiry of the first node.

### 8.6. Delay

The overall time it takes for packets to arrive at their destination is referred to as delay. WBAN may track any critical human body parameter, such as the electrical activity of the heart. As a result, in time-critical applications, delay must be investigated to ensure that data arrives at the sink on time.

Table 4 shows a comparison of the solutions discussed in the literature review section based on the performance factors holding above.

Clustering-based routing techniques have shown to be more suitable for WBAN applications than crosslayer and thermal-aware routing techniques since then. In a clustered-based system, data is sent to the base station through cluster heads in their designated time slots, reducing energy consumption and increasing the stability period.

- Further challenges: different cluster-based, energy-efficient, and reliable routing algorithms have been developed to improve the maximise throughput, network stability and achieve longevity in WBAN network operations. Still, a number of issues and concerns must be addressed by the research community, including several solutions ignore energy conservation throughout the network deployment, network organisation, and internode communication phases [29]
- The forwarder node selection criteria and the optimal amount of relay nodes are ineffective, and the load is not evenly distributed among sensor nodes [28]
- In terms of reliability, energy consumption, routing overhead, and scalability, selecting a forwarder node in round by round is inefficient. As a result, a static adaptive clustering strategy must be devised
- When packets are dropped by a node to retain more residual energy for desiring a forwarder node, this is known as a selfish node assault. As a result, a trust-based provision is required to improve network reliability [87]
- The expected transmission count (ETX) and routing link metrics are significant elements that are not examined in existing clustering-based techniques [88]
- Throughput is another important factor to consider, and the location of the sink can have a big impact on it [89]

As a result of the explanation above, it is evident that reliability and energy efficiency are major issues in resource-constrained WBANs. As a result, it is necessary to develop reliable and energy-efficient routing approaches that may improve the reliability and network stability while taking into account the particular features and requirements of resource-constraint WBANs in critical applications.

RETRACTED

## 9. Conclusion

WBAN (wireless body area network) is a subset of wireless sensor networks (WSNs) with its own set of characteristics due to resource constraints and application scope. We presented an overview of WBAN applications and architecture in this post, highlighting current research topics and challenges. Because sensor nodes in WBANs have limited resources, energy efficiency and reliability are critical considerations. We assessed the present state-of-the-art solutions in WBANs for energy efficiency and reliability, identifying their strengths and drawbacks. We also identified several performance characteristics that must be considered when creating and evaluating WBAN solutions. Finally, we identified a number of issues and obstacles in terms of energy efficiency and reliability in WBANs that need to be addressed further in the development of new WBAN solutions. As part of our ongoing study, we have presented a novel energy-efficient and reliable routing strategy to improve the stability period and network lifetime in WBAN. In this research work, the emerging technology like edge computing, Fog computing, and AI techniques is not discussed. We aim to work on these limitations in our future research findings with the research community via future publications.

RETRACTED

## Figures and Tables

**Figure 1:** Generic structure of WBAN.

**Figure 2:** Communication architecture of WBAN.

**Figure 3:** Classification of energy efficient routing protocols in WBAN.

**Table 1:** Commonly used abbreviations.

WBAN	Wireless body area network
BS	Base station
ECG	Electrocardiography
WSN	Wireless sensor network
BER	Bit error rate
EMG	Electromyography
SAR	Specific absorption ratio
QoS	Quality of service

**Table 2:** Key consideration of WBAN applications.

Application type	Sensor node	Type of sensor	Bandwidth (Hz)	Accuracy (bits)	Data rate	Duty cycle % per time	Power consumption	QoS	Privacy
In-body application	Glucose sensor	Strip-base	0-50	16	Few kbps	<1%	Very Low	Yes	High
	Pacemaker	Accelerometer	0-500	12	Few kbps	<1%	Low	Yes	High
	Endoscope capsule	A pill and contains a tiny camera	..	..	>2 mbps	<50%	Low	Yes	Medium
On-body medical application	ECG	Skin/chest electrodes	100-1000	12	192 kbps	<10%	Low	Yes	High
	EMG	Skin electrodes	0-10000	16	1.536 mbps	..	Low	..	..
	Temperature	Temperature probes or skin patch	0-1	8	56 kbps	..	Low	..	..
	SpO2	Pulse oximeter	..	..	32 kbps	<1%	Low	Yes	High
	Blood pressure	Arm cuff-based monitor	0-1	8	<10 bps	<1%	High	Yes	Medium
On-body nonmedical application	Music for headsets	Sound	..	..	1.4 mbps	High	Very high	Yes	Low
	Forgotten things monitor	Monitor	..	..	256 kbps	Medium	Low	No	Low
	Social networking	Mixed sensor	..	..	<200 kbps	<1%	Low	No	High

**Table 3:** Requirement of WBANs.

Applications	Bit rate	BER	Delay
Drug delivery	<16 kbps	<10^−10^	<250 ms
ECG	3 kbps	<10^−10^	<250 ms
EMG	120 kbps	<10^−10^	<250 ms
Glucose level monitoring	<1 mbps	<10^−10^	<250 ms
Temperature	120 bps 56 kbps	<10^−10^	<100 ms
SpO2	150 kbps	<10^−10^	<100 ms
Audio streaming	1 mbps	<10^−10^	<20 ms
Video streaming	<10 mbps	<10^−10^	<100 ms
Voice	50-100 kbps	<10^−10^	<100 ms

**Table 4:** Performance analysis of existing schemes.

Schemes/solutions	Characteristics						
	No. of dead nodes	Packets sent to sink	Packet dropped ratio	Packet received at sink	Thermal aware approach	Network stability period	Delay
IM-SIMPLE [1]	Medium	High	Medium	Medium	No	Medium	Medium
DARE [14]	Medium	High	Medium	Medium	No	Medium	High
M-ATTEMPT [23]	High	Medium	Medium	Medium	Yes	Low	Medium
SIMPLE [28]	Medium	Medium	Medium	Medium	No	Medium	Medium
FEEL [29]	Medium	High	Low	High	No	High	Medium
TARA [56]	High	Low	High	Low	Yes	Low	High
LTR [57]	High	Low	High	Low	Yes	Low	High
ALTR [57]	High	Medium	Medium	Medium	Yes	Low	Medium
LTRT [58]	Medium	High	Low	High	Yes	Medium	Medium
RE-ATTEMPT [59]	Medium	High	Medium	Medium	No	Medium	Low
M^2^E^2^ [61]	Medium	High	High	Medium	Yes	Medium	Medium
CO-LAEEBA [79]	Low	High	Low	High	No	High	Low
WASP [85]	High	Medium	Medium	Medium	No	Low	Low
CICADA [86]	Medium	High	Low	High	No	Medium	Medium
ERRS	Medium	High	Low	High	No	High	Low

RETRACTED

## Data Availability

No data were used to support this study.
